# Megakaryocytic dysfunction in immune thrombocytopenia is linked to autophagy

**DOI:** 10.1186/s12935-019-0779-0

**Published:** 2019-03-15

**Authors:** Rui-jie Sun, Ning-ning Shan

**Affiliations:** Department of Hematology, Shandong Provincial Hospital Affiliated to Shandong University, 325 Jing Wu Rd, Jinan, 250021 Shandong People’s Republic of China

**Keywords:** Autophagy, Megakaryopoiesis, ITP

## Abstract

Immune thrombocytopenic purpura (ITP) is a multifactorial autoimmune disease characterized by both increased platelet destruction and/or reduced platelet production. Even though they are detected in ≤ 50% of ITP patients, auto-antibodies play a pivotal role in the pathogenesis of ITP. Recent experimental and clinical observations have revealed abnormal autophagy in ITP patients. Autophagy is a catabolic process responsible for the elimination and recycling of cytoplasmic constituents, such as organelles and macromolecules, in eukaryotic cells. Additionally, it triggers cell death or promotes cell survival following various forms of stress, and maintains the microenvironment and stemness of haematopoietic stem cells. The role of autophagy in megakaryopoiesis, thrombopoiesis, and platelet function is slowly being uncovered. The abnormal autophagy in ITP patients may be caused by deletion of autophagy-related genes such as ATG7 and abnormal signalling due to overexpression of mTOR. These changes are thought to affect markers of haematopoietic stem cells, such as CD41 and CD61, and differentiation of megakaryocytes, ultimately decreasing the function and quantity of platelets and leading to the onset of ITP. This review highlights recent evidence on the essential role played by autophagy in megakaryopoiesis, megakaryocyte differentiation, thrombopoiesis, and platelet production. It also discusses the potential of targeting the autophagy pathway as a novel therapeutic approach against ITP.

## Introduction

Autophagy is a highly conserved biological process in eukaryotic cells. It is involved in cell development, starvation adaptation, intracellular quality control, tumour suppression, ageing, innate immunity, and other processes [1, 2]. However, both insufficient and excessive autophagy can lead to pathological conditions [3]. In recent years, experimental and clinical evidence has associated perturbations of normal autophagy processes with a number of neoplastic and autoimmune diseases [4], such as myelodysplastic syndrome (MDS) [5], chronic myelogenous leukaemia (CML) [6], systemic lupus erythematosus (SLE) [7], rheumatoid arthritis (RA) [8], multiple sclerosis (MS) [9], and aplastic anaemia (AA) [10]. In another autoimmune disease, immune thrombocytopenic purpura (ITP), autophagy plays an important role in maintaining the stemness and the microenvironment of haematopoietic stem cells [11]. Thus, on the one hand, autophagy ensures the proper differentiation of haematopoietic stem cells into megakaryocytes. On the other hand, at an early stage of megakaryocyte differentiation, induction of autophagy by inducer rapamycin or inhibitor bafilomycin A1 appears to impede megakaryocyte maturation, reduce platelet formation in bone marrow, and affect platelet function [12]. Further on, in mature megakaryocytes, autophagy deficiency induces abnormal platelet activation and function, without changing platelet number and size [13]. Accordingly, it appears that an abnormal level of autophagy causes different effects during distinct stages of cell differentiation [13]. Recently, autophagy has been demonstrated to be indispensable for normal megakaryopoiesis and platelet function in animal models with lineage-specific deletion of autophagy-related genes (ATGs) [14]. Excessive expression of mammalian target of rapamycin (mTOR) was reported in diseases related to megakaryocytes such as ITP, in which it inhibited autophagic activity and affected the differentiation of haematopoietic stem cells into megakaryocytes, the formation of megakaryocytes, and platelet function [15] Improving our understanding of autophagy will likely result in new therapeutic methods aimed at inducing autophagy-related proteins to counteract megakaryocyte/platelet disorders in clinical conditions. For example, induction of autophagy by rapamycin has already exhibited substantial therapeutic benefits in patients with ITP [16].

## Autophagy

Autophagy, also called autophagocytosis, is a self-eating [17] and stress-induced catabolic process that delivers defective organelles and cytoplasm to the lysosome [18], and eventually forms the autolysosome. And this process also named the autophagy-lysosomal pathways (ALPs) [17]. The autophagy cytoplasmic quality control system supports the function and survival of different types of cells in most tissues of the body, for example, it provide the capability to quickly remove toxic waste and to repurpose unnecessary material [18]. Autophagy is upregulated in response to starvation, nitrogen deprivation, extra environmental and oxidative stresses, toxin and infection, DNA damage, and is downregulated in response to rapamycin treatment (Fig. 1). Based on different transport pathways and substrates in mammalian cells, autophagy can be divided into several distinct forms termed macroautophagy, microautophagy, chaperone-mediated autophagy (CMA) [19], mitophagy and aggrephagy [17], which are induced by similar stimuli and provide protection against most of diseases. Amongst these types, macroautophagy has been the most extensively studied. It is the major core of the ALPs and can be further divided into pexophagy, mitophagy, and non-selective autophagy [20].

**Fig. 1:** Autophagy signalling pathways. As a complex multi-step process, autophagy is accompanied by the distinct sets of autophagy-related genes mediating key steps from autophagic induction to vesicle fusion and autophagosome breakdown. Stimuli such as immune signals, starvation, growth factor deprivation, infection, and oxidative stress have been demonstrated to induce autophagy. These stresses inhibit the mTOR kinase and consequently induce autophagy. Autophagy initiation is directly regulated by the serine/threonine protein kinases ULK1/2 complex, which then forms a complex with beclin 1. Subsequently, an isolation membrane envelops cytoplasmic constituents, and elongates through the action of two ubiquitin-like conjugation systems to form a double-membrane autophagosome. Autophagosomes fuse with lysosomes to form autolysosomes, and finally the vesicle contents are degraded

At different stages of the autophagy pathway, a variety of ATG protein act as different function. For example, E1 enzyme ATG7 can activate autophagosome by two ubiquitin-like conjugated systems, UB1 protein ATG12 and ATG8 [21]. Briefly, autophagy consists essentially of a survival mechanism that is activated under adverse conditions to maintain cell integrity. However, paradoxically, it is also involved in a particular form of cell death called autophagic cell death or type II cell death [6].

### Autolysosome and autophagy signalling

For macroautophagy, targeted cytoplasmic components undergo sequestration by endoplasmic reticulum membrane vesicles to formed phagophore (Fig. 1). Then the phagophore expand and close to form an autophagosome, a double-layered vesicle that isolates the cytoplasmic material. By fusing to a lysosome, the autophagosome turns into an autolysosome and degrades its content through acidic hydrolysis. Finally, the captured material and inner membrane are degraded or recycled [15, 22]. Micro-autophagy, to some extent, resembles macro-autophagy, but the contents of micro-autophagy are directly consumed by lysosomes [23]. Chaperone-mediated autophagy operates through the hsc70-containing complex, with has high selectivity for specific substrates [24].

The canonical autophagy pathway consists of more than 34 autophagy-related genes (ATGs), originally identified in yeast. And nearly half of them are conserved in mammals [25]. The complete process of autophagy including activation, target identification, autophagosome formation, lysosome fusion, and degradation, is driven by defined ATG proteins [26]. For example, ATG1–10, 12,13,14, 16,17,18, 29, and 31 are essential for the formation of canonical autophagosomes [27]. Here, we describe each of these steps individually, accompanied by instruction for the major genes associated with each sub-process.

#### Initiation

Under the stimulus mentioned above, a double-membrane structure called phagophore emerges [17]. Two major complexes, ULK complex and PI3K complex, are recruited to the phagophore assembly site (PAS). The PAS is a single-site structure close to the yeast vacuole membrane, where almost all Atg proteins aggregate to form the isolation membrane and autophagosomes [25]. The former is consists of Unc-51 like autophagy activating kinase 1/2 (ULK1/2, ATG1 in yeast)—ATG13-ATG101-FAK family kinase-interacting protein of 200 kDa (FIP200), also known as RB1CC1 (RB1 inducible coiled-coil 1) [18]. The ULK complex is activated in biochemically by inactivation of its negative regulator mammalian target of rapamycin complex1 (mTORC1) and other signaling pathways, such as its positive regulator activated by 5-AMP protein kinase (AMPK) [28–30]. The active ULK complex is enriched at the presumptive autophagosome assembly sites, where it engages downstream regulatory machinery including the autophagic class III phosphatidylinositol 3-kinase (PI3K) [18]. The latter contains Beclin1, (BECN1; ATG6 in yeast), Beclin1, VPS34 (the catalytic PIK3C3 subunit), VPS15, ATG14L (also known as Barker), and NRBF2 [18]. The PI3K complex bind to Beclin 1 and antagonize the interaction of Beclin 1 with Vps34 [31, 32]. PI3K also produce phosphatidylinositol 3-phosphate (PtdIns [3] P, PI3P) to concentrate at the surface of the phagophore and recruit other ATGs to the PAS to promote the formation of the autophagosome [33].

The conserved nutrient-sensing serine/threonine kinase mTOR plays a vital inhibitory role in the regulation of autophagy. mTOR forms two distinct complexes, which vary both in their subunit components and function. Thus, mTOR complex (mTORC) 1 is responsible for autophagy regulation [34], especially during nuclear division, cell cycle progression, and T cell differentiation and metabolism [35]. Besides, it is also important during the early and late stage of megakaryocyte development and maturation [36]. Autophagy is initiated through inactivation of mTORC1 following hypoxia, starvation and pharmacological treatment with rapamycin [37]. In contrast, mTORC2 is not a direct autophagy regulator [38], as its main task is to control cell size and cell death [35].

Other autophagy pathways have also been identified; these include the Ras/cAMP-dependent protein kinase pathway [39], the lKB1-AMPK pathway [40], and Bcl-2, which is an anti-apoptotic protein that interacts with beclin 1 to inhibit autophagy [31].

#### Elongation

The formation of autophagosomes is regulated mainly via two ubiquitin-like (Ubl) conjugation systems: Atg8 (LC3)-PE (phosphatidy lethanolamine) system and ATG5-ATG12-ATG16 (L) system [41]. Both systems are required for decorating the expanding phagophore [42, 43]. The first system cleaves microtubule associated protein 1 light chain 3 (LC3, the mammalian orthologue of yeast ATG8) that is activated by ATG7 into LC3-I by ATG4B, and then cleaves LC3-I into LC3-II and transferred to the E2 conjugating enzyme ATG3 by ATG7 [44]. Finally, ATG8 is conjugated with the target lipid PE to form ATG4B-ATG3-ATG7-LC3 (ATG8) complex [44, 45]. The second system is crucial for the elongation of the pre-phagosomal structure and aid to the formation of LC-3II [46]. The recruitment and localization of LC3 plays a vital role in autophagosome formation and also act as an important marker to evaluate the level of autophagy [47, 48]. When activated, ATG12 is transferred to the E2 enzyme ATG10 and then binds to an internal lysine of its substrate protein ATG5, ATG12-ATG5 bind to a coiled-coil protein ATG16 to form an E3-like multimer complex [42, 49], which then binds to ATG3 and promotes autophagosome nucleation. Meanwhile, activated ATG3 covalently binds to LC3, which is lipidated by ATG16L and associates with the autophagosome membrane with PE [42].

#### Fusion and breakdown

After the forming of bubble-like autophagosome, the ATG12-ATG5-ATG16 (L) complex is released to the cytoplasm. However, ATG8-PE complex follows the autophagosome into the vacuole and cleaves by ATG4 to release ATG8 to lysosomal for degradation [50]. The autophagosome can move bidirectionally along microtubules via the aid of motor proteins and then fusing with lysosome to form autolysosome by the aid of multiple protein complexes, such as soluble NSF attachment protein receptors (SNAREs) [51–53]. The autophagosomes are then digested by lysosomal enzymes. The next, the single membrane of the autophagosome is broken down to recycle cellular molecules. Two conserved components involved in the process of breakdown were identified in yeast, ATG15 and ATG22 [21]. ATG15 is involved in the degradation of the inner vesicle [54, 55]. While the intact vacuolar membrane protein ATG22 is responsible for the transport of small molecules, such as amino acids and other small molecules, back to the cytoplasm for protein synthesis and cell function maintenance during autophagy [56].

### The role of autophagy in autoimmune disease

Under physiological conditions, autophagy not only regulates core cellular processes such as survival of immune cells and cytokine-dependent inflammation during endogenous distress [57], but it also plays a primordial role in controlling intracellular pathogens [20]. A number of immune processes including pathogen recognition and destruction [58], antigen presentation [59], lymphocyte development and function [60], the humoral immunity process [61], and inflammatory regulation [20] are highly dependent on autophagy. Moreover, evidence indicates that autophagy participates in the activation and proliferation of T and B lymphocytes [7], as well as the mechanism dictating survival of B cells [62]. Besides, under pathological conditions, autophagy becomes abnormal as it ensures an adequate response to different extracellular and intracellular forms of stress [63, 64]. Hence, autophagy provides a critical protective mechanism for the body.

Abnormalities in the autophagic cascade pathways are potential risk factors for numerous autoimmune diseases [65]. Consequently, understanding autophagy and misregulation of the process has become an important goal in autoimmune and chronic inflammatory disease [66]. Although the precise mechanisms by which abnormal autophagy functions make the host more susceptible to continuous inflammation remain unclear, genome-wide association studies have confirmed that multiple changes in autophagy-related genes are related to the susceptibility to tissue damage in systemic lupus erythematosus [67] and inflammatory bowel disease [68]. Moreover, autophagy’s role in regulating the survival time of adaptive immune cells has been demonstrated in rheumatoid arthritis [8] and multiple sclerosis [9].

#### SLE

As a core pathogenic contributor affecting both innate and adaptive immunity, autophagy has been implicated in multiple malfunctions relevant to SLE [69], including removal of dead cells, clearance of intracellular DNA and RNA, control of the activation and survival time of B cells and T cells, and regulation of type I interferon (IFN) responses [70]. Currently, the consensus is that autophagy is higher in SLE [71]. A possible role of ATG7 and ATG5 in modulating SLE pathology has been examined in a murine model of SLE. Moreover, drugs regulating autophagy, including rapamycin, hydroxychloroquine, and P140 peptide, have been observed to provide beneficial effects in mouse and patients with SLE, emphasizing that resetting autophagy flux may be an important therapeutic target for this autoimmune disease [72].

#### Crohn’s disease

Although the underlying mechanism has remained incompletely understood, ATG16L1 deletion has been demonstrated to be associated with disease susceptibility in mouse model of Crohn’s disease [68]. High amounts of the proinflammatory cytokine IL-18 were released from Atg16L1-deficient macrophage, strengthening the link between Atg16L1 and inflammasome activation [68]. And relevant studies have reported that ULK1 gene increases susceptibility to Crohn’s disease [73], confirming the relationship between gut inflammation and autophagy.

#### MS and RA

Autophagy interferes with survival of lymphocyte, antigen-presenting and antigen-responsive cells in MS and RA [66]. In patients with MS, the expression of ATG5 was up-regulated in T cells infiltrating inflammatory sites [9]. In RA, ATG5 interfered with presentation of citrullinated peptides [8], and RA patients have significantly lower levels of LC3 and Beclin-1 [66].

## Autophagy and immune thrombocytopenia

Platelets are small anucleate cytoplasmic fragments derived from megakaryocytes, the primary physiological role is to mediate thrombosis and hemostasis [74]. Activated platelets secrete microparticles which accelerate the plaque formation by providing a new prothrombotic interface and promoting the deposition of fibrin and other blood cells at the site of thrombus formation [75, 76]. Ouseph et al. has demonstrated that basal level of autophagy process is essential for normal functioning of platelets activation and aggregation. And they further showed that platelet specific deletion of Atg7 can cause a decrease granule cargo packing ex vivo [77]. In another study, they demonstrate that starvation induced substantial autophagy (above basal level), characterized by decreased platelet aggregation, reduced calcium mobilization and granule secretion, as well as decreased adhesion to immobilized fibrinogen and eventually increased bleeding time [78]. Autophagy antagonize platelet activation by clearance certain potentially ubiquitinated proteins. These studies collectively demonstrated that basal level of autophagy in platelet is obligatory for aggregation, activation, hemostasis, and thrombosis [77, 78].

ITP is a common autoimmune-mediated bleeding disease, in which platelet membrane proteins become antigenic, stimulate the immune system to produce antibodies, and eventually result in thrombocytopenia [15]. About 50% of ITP patients have auto-antibodies that not only destroy platelets, but also impair megakaryocyte maturation and platelet production by the bone marrow [79]. In one study, a comparison of ITP mice and normal mice revealed that the former were characterised by higher frequencies of immature megakaryocytes/platelets and corresponding progenitor cells, as well as increased phagocytosis. These findings could explain the decrease in peripheral blood platelet counts observed in ITP patients [80]. McMillan and co-workers [79] previously described defective megakaryopoiesis in C-ITP (chronical immune thrombocytopenia) patients. They showed that, the addition of anti-platelet antibodies to normal megakaryocytes in liquid culture led to impaired megakaryocyte proliferation and abnormal ploidy distribution. Recently, Cao et al. [14] used an ATG7 haematopoietic conditional knockout mouse model to show that core autophagy machinery was important for normal megakaryopoiesis and platelet function. Thus, in ITP patients, the loss of autophagy prevents megakaryocyte formation and differentiation, negatively affects thrombopoiesis, and results in larger but fewer platelets, ultimately severely impairing platelet production [14]. Finally, Ouseph et al. [77] have demonstrated that autophagy is involved in the maturation of megakaryocytes and represents an important pathological condition in ITP patients (Fig. 2).

**Fig. 2:** Recent evidence describing the pathogenesis of autophagy in ITP. Lineage-specific deletion of ATG in haematopoietic stem cells (HSCs) impairs megakaryopoiesis in the bone marrow. The enhanced expression of mTOR on the surface of megakaryocytes decreases the extent of autophagy. A close connection between the above steps leads to fewer platelet counts in the bone marrow and peripheral blood, as well as abnormal haemostasis

### Impaired autophagy affects the differentiation of haematopoietic stem cells into megakaryocytes

During haematopoiesis, haematopoietic stem cells give rise to two lineages, a common lymphoid progenitor capable of producing lymphocytes, and a common myeloid progenitor with developmental potential restricted to granulocytes/monocytes, basophils, eosinophils, erythroid cells, and megakaryocytes [81]. Autophagy plays an important role in maintaining the stemness and the microenvironment of haematopoietic stem cells [11]. Autophagy is also required for self-renewal and differentiation of CD34+ CD133+ cells, and it serves as an adaptive stress response mechanism in haematopoietic stem and progenitor cells [82, 83]. Although the role of autophagy in cell differentiation remains ill-defined, there is some evidence that it might control differentiation processes [84–86]. Deletion of ATG7 in haematopoietic stem cells results in failure to maintain such a pool of cells and is implicated in the development of myeloid malignancies [87]. Thus, ATG7 haematopoietic conditional knockout mice develop severe anaemia. Furthermore, ATG7-erythrocytes accumulate damaged mitochondria with altered membrane potential, leading to cell death. Mitochondrial damage caused by ATG7 deficiency leads also to severe lymphopaenia, when followed by apoptosis in mature T lymphocytes of SLE patients [88]. The ATG- mouse model used by Cao et al. [14], displayed abnormal megakaryocyte differentiation and proliferation, as well as thrombopoiesis, ultimately resulting in failed platelet production and haemostasis. CD41 and CD61 are the two markers of megakaryocytic cells; the percentage of CD41+ CD61+ cells was reduced in ATG7- bone marrow cells, and was associated with increased apoptosis and necrosis [14].

When autophagy was inhibited by bafilomycin A1 or induced by rapamycin in cells, the similar result was observed that significant decrease in high ploidy megakaryocytes, a reduction of CD41 and CD61 co-expressing cells, and less proplatelet or platelet formation [12]. However, when autophagy was altered in mature megakaryocytes, there was no significant change in proplatelet formation, which was consistent with normal platelet counts, megakaryocyte numbers [12]. In summary, the data indicate that either upregulated or inhibited autophagy in the early stage of megakaryopoiesis suppresses megakaryopoiesis and thrombopoiesis [12]. Cell cycle analysis revealed that ATG7 deficiency caused apoptosis and fewer diploid or polyploid progenitor cells [14]. In summary, autophagy is required for the survival of haematopoietic stem (CD34+) cells and their differentiation into megakaryocytes.

### Abnormal autophagy affects the differentiation of megakaryocytes into platelets

Haematopoiesis, megakaryopoiesis, megakaryocyte differentiation, and thrombopoiesis are successive maturation processes that include polyploidization, development of an extensive internal membrane system, formation of proplatelet processes, and finally the organized release into blood vessels, which undergo repeated abscissions to yield circulating platelets [89, 90]. Mature megakaryocytes can be identified by specific cell surface markers including CD41, CD61 (integrin αIIbβ3), CD42 (glycoprotein Ib), and glycoprotein V. Recently, ATG7 knockout mouse model has demonstrated the indispensable role of autophagy for normal megakaryopoiesis and platelet function, both in hematopoietic conditions or in megakaryocyte and platelet conditions [14, 77]. Various ultrastructural abnormalities of ITP megakaryocytes have been reported; these include altered vacuoles, markedly expanded demarcation membrane systems, mitochondrial swelling, and the emperipolesis of other marrow cells. Importantly, platelet morphology and production can be affected by abnormalities at any stage of megakaryocyte production [91]. Disruption of the autophagic flux leads to impairment of platelet aggregation and adhesion. The result indicates the important role of ATG7 in platelet activation and haemostasis [14]. Houwerzijl et al. [92] reported ultrastructural abnormalities compatible with (para-) apoptosis in bone marrow megakaryocytes, implying that megakaryocyte damage could reduce platelet production in ITP. Specifically, the study showed quantitative and qualitative abnormalities in proplatelet production in the presence of ITP plasma; this may reveal new mechanisms contributing to the development of thrombocytopenia in ITP [10].

### Autophagy target treatment for immune thrombocytopenia

Traditional first-line treatments of ITP, such as corticosteroid, intravenous immunoglobulin and intravenous anti-D, are successful, but do not usually result in long-term remission. Second- and third-line therapies, including splenectomy, Rituximab, immunosuppressants, and thrombopoietin-A, are often effective, and particularly the first two may increase platelet counts on the long term. However, many patients are unfit for splenectomy and the therapy above may cause serious side effects, particularly following prolonged treatment. Thus, it is paramount to explore novel treatments for ITP [80, 93, 94].

As emerging roles of autophagy in megakaryopoiesis, thrombopoiesis, and platelet function have been revealed in patients with thrombocytopenic disorders, insights into signalling pathways may guide future research in this field. The rapamycin-sensitive protein mTORC1 plays an important role in the regulation of T cell differentiation and metabolism [95], and it may represent a new therapeutic target for ITP. mTOR inhibitors rapamycin and WYE-354 (which can induce autophagy) promote autophagosome formation and induce autophagy. Moreover, they display protective and beneficial effects on murine lupus nephritis [96, 97] and patients with lupus nephritis [98]. Unfortunately, the characteristic poor water solubility of rapamycin limits its clinical application. A more water-soluble drug against mTOR, sirolimus (CC1779), has been approved for the clinical treatment of renal cell carcinoma, and other similar drugs have been approved for the reduction of renal transplant rejection and clinical treatment of coronary artery stenosis [99]. Another mTOR inhibitor, AZD8055, is used as a spare drug treatment for SLE [100]. AZD8055 is taken orally, and its mode of action involves inhibiting the activation of mTORC1 and mTORC2. Therefore, these drugs can reduce the risk of tumours in SLE patients [98]. The clinical application of autophagy therapy for SLE may be enlightening for the future therapy of ITP. In vitro experiments with MKs from mutant mice showed that rapamycin induced autophagy and decreased the size and ploidy of megakaryocytes [13]. Moreover, results from a clinical trial on ITP patients suggest that rapamycin is an effective treatment against immune-induced thrombocytopenia [16]. Therefore, targeting autophagy may yield a promising approach for thrombocytopenic diseases. Other studies have revealed that low-dose DAC (Decitabine) (10 nM) could significantly increase the number of mature polyploid (≥ 4 N) megakaryocytes [101]. Finally, lapatinib treatment induces ATG-mediated autophagy and megakaryocytic differentiation in K562 cells of CML [102]. In summary, the above autophagy-targeted therapies might lead to novel clinical treatments in ITP patients.

## Conclusion and future perspectives

In this review, we summarized the limitations of current therapies and highlighted new treatments for ITP. The important role of autophagy in autoimmune diseases provides a new opportunity for understanding the pathogenesis of ITP. In particular, knowledge of the mechanism underlying abnormal autophagy in immature megakaryocytes may be important for the treatment of ITP patients. Similarly, autophagy induction may offer a novel therapeutic strategy against ITP or immune diseases, especially within the context of individualized treatment and disease control.

However, the study of Liu et al. demonstrated that the plasma in ITP patients induces autophagy and suppresses apoptosis [103]. And the inhibition of autophagy may be a novel treatment in further investigation. This conclusion deserves further research. For example, current results need more case validation analyses, functional verification assays and larger population-based studies to confirm [103]. And this conclusion is in contrast to our treatment of ITP autophagy induced by rapamycin. It could be interesting to explore this point and explained the role of autophagy in ITP as a balance between hyperactivity and inhibition in future.

In general, future research will benefit from focusing on targeted regulation of autophagy and related receptors, recognition mechanisms, and possible biomarkers. These will complement additional more in-depth studies on existing treatments for autophagy-based disorders.

## Abbreviations

ITP: immune thrombocytopenia
ATG: autophagy related genes
mTOR: mammalian target of rapamycin
MDS: myelodysplastic syndrome
CML: chronic myelogenous leukaemia
SLE: systemic lupus erythematosus
RA: rheumatoid arthritis
MS: multiple sclerosis
AA: aplastic anaemia
